# Simvastatin Inhibits Endometrial Cancer Malignant Behaviors by Suppressing RAS/Mitogen-Activated Protein Kinase (MAPK) Pathway-Mediated Reactive Oxygen Species (ROS) and Ferroptosis

**DOI:** 10.1155/2022/6177477

**Published:** 2022-10-14

**Authors:** Dan Zhou, Qiuhua Wu, Huajuan Qiu, Mi Li, Yanqin Ji

**Affiliations:** Department of Gynaecology, Huizhou Central People's Hospital, Huizhou, Guangdong 516008, China

## Abstract

This paper was designed to explore the function of simvastatin as a chemotherapeutic drug on the endometrial cancer (EC) cell proliferation, invasion, and ferroptosis. Firstly, a number of *in vitro* experiments were conducted to determine the impact of different treatments of simvastatin on the Ishikawa cell invasion, proliferation, and colony formation. The concentration of DCFH-DA-labeled reactive oxygen species (ROS) in cells was assessed by flow cytometry. Enzyme-linked immunosorbent assay (ELISA) was performed to examine the intracellular contents of Fe^2+^, malondialdehyde (MDA), and glutathione (GSH). Additionally, Western blot was utilized to measure the expression level of RAS/mitogen-activated protein kinase (MAPK)-related proteins and ferroptosis-related proteins in cells. The results showed that simvastatin at 10 *μ*M and 15 *μ*M apparently suppressed the proliferation of Ishikawa cells, colony formation, and invasion ability of Ishikawa cells, and upregulated the level of MDA and ROS, but downregulated the level of GSH. Besides, 10 *μ*M and 15 *μ*M of simvastatin promoted cell ferroptosis (up-regulation of Fe^2+^ and TRF 1 protein level; down-regulation of SLC7A11 and FPN protein level) and lowered the RAS, p-MEK, and ERK protein level. Furthermore, experiments also revealed that the inhibitory effects of simvastatin on Ishikawa cell proliferation, colony formation, and invasion, as well as the promoting effects on oxidation and ferroptosis were reversed. All in all, simvastatin reduces the RAS/MAPK signaling pathway to inhibit Ishikawa cell proliferation, colony formation, and invasion, and promote cell oxidation and ferroptosis. This paper demonstrates the potential of simvastatin as a new anticancer drug for EC.

## 1. Introduction

As one of the three most prevalent malignancies of the female reproductive system, endometrial cancer (EC) is also the sixth most common malignant tumor in women. Recent years have witnessed the rapidly increased incidence of EC due to declined birth rate, climbed aging population, changed lifestyle changes, and other factors [1, 2]. In 2018, 382,000 new cases and 89,000 deaths were reported globally, with 12% of new cases reported in China [2]. Approximately one-fifth of EC cases are characterized by high risk and poor prognosis, for instance, the 5-year overall survival rate is less than 20% in EC patients with distant metastasis [3, 4]. The effectiveness of total hysterectomy for EC is unsatisfactory [5], and new therapies are needed to further improve the survival rate of patients.

Ferroptosis is known as a regulated type of iron-dependent cell death as a result of a buildup of lipid-based reactive oxygen species (ROS). As a recently identified type of regulated cell death, ferroptosis has new biological targets and pathophysiology features [6]. ROS buildup serves as one of the characteristics of ferroptosis. During ferroptosis, transferrin receptor 1 (TRF1) expression and ferritin degradation are both significantly regulated by ROS-induced autophagy. Some research studies have revealed that ferroptosis is linked to various diseases, such as ischemic organ damage, neuro-degeneration, liver and pulmonary fibrosis, autoimmune diseases, mycobacterium tuberculosis-induced tissue necrosis, smoking-related chronic obstructive pulmonary disease, and cancers [7, 8]. The female reproductive system has a special relationship with iron; iron disorders and iron-mediated cell deaths are closely associated with a variety of endometrium-related diseases including endometrial hyperplasia, recurrent implantation failure, and endometriosis [9]. The research on ferroptosis in EC is, however, scant. Wang et al. stated that the down-regulation of PTPN18 could significantly stimulate the production of ROS and inhibit EC cell proliferation, and through the p-p38/GPX4/xCT axis, PTPN18 could induce ferroptosis [10]. Bioinformatics analysis by Yin et al. revealed that multiple ferroptosis-related genes could serve as predictors for the prognosis of EC patients [11].

Statins, as 3-hydroxy-3-methylglutaryl coenzyme A (HMG-CoA) reductase inhibitors, by lowering the level of low-density lipoprotein cholesterol (LDL-C), are commonly adopted to improve the morbidity and mortality of cardiovascular patients [12]. In addition, statins have anticancer effects, and their anticancer effects are associated with the regulation of growth factor receptors and cholesterol-dependent signaling in tumor cells [13]. Specifically, statins can suppress HMG-CoA reductase, deplete mevalonic acid and its downstream products, and ultimately induce tumor cell apoptosis [14]. Compared with the other statins, simvastatin shows the best lipophilicity and therapeutic effect [15]. Simvastatin can enter cells through the organic anion transporter (OATP1B1) to interrupt mevalonate pathway and inhibit LDL-C production [16]. In vitro experiments confirmed that simvastatin affected the migration, proliferation, and survival of various cancer cells [17]. Simvastatin has been shown in numerous in vitro experiments to slow the spread of cancer and lower mortality in individuals with pancreatic, stomach, breast, and lung cancers. [18].

The effects of simvastatin on the progression of EC remain unclear. Therefore, we investigated the molecular mechanism of simvastatin on Ishikawa cells and the effect of treating Ishikawa cells with RAS activator (ML-098) by in vitro experiments. The results showed that simvastatin exerted therapeutic effects on EC by reducing RAS/MAPK signaling pathway activity, suppressing the invasion, clone formation and proliferation of Ishikawa cells, and promoting cell oxidation and ferroptosis. Therefore, we hypothesized that simvastatin is a promising drug option for the therapy of EC. Our experiments confirmed this hypothesis.

## 2. Materials and Methods

### 2.1. Cell Culture and Treatment

EC cells (Ishikawa) were grown in a high-glucose DMEM medium that contained 10% fetal bovine serum (FBS) and 1% penicillin-streptomycin. And the medium was placed in an incubator with 5% of CO_2_ at 37°C. Subsequently, Ishikawa cells were treated with simvastatin (5 *μ*M, 10 *μ*M, and 15 *μ*M) for 72 h [19], or with simvastatin + RAS agonist (0.5 *μ*M) for 72 h [20]; the cultured cells without treatment acted as a control.

### 2.2. MTT Assay

As previously mentioned, the MTT assay was carried out [9]. In brief, trypsin (Beyotime, China) was adopted to digest the cells in the logarithmic phase for the preparation of cell suspension. Then, a 96-well plate was introduced with 100 *μ*L cell suspension at 3000 cells per well and then placed in an incubator at 37°C for cell adhesion. Subsequently, cells were then treated with different reagents for 72 hours following the experiment requirements. According to the MTT kit (Beyotime, China) instructions, the proliferation of cells before and after treatment was tested, respectively. To be specific, 10 *μ*L (5 mg/ml) of cell suspensions was supplemented to the plate and incubated for 4 hours at 37°C. After adding 100 *μ*L of Formazan dissolving solution, the incubation was continued until the precipitate was fully dissolved. Finally, we use a microplate reader (Thermo Fisher Scientific, Waltham, USA) to detect the absorbance value at 570 nm and calculate the cell viability, and we carried out the experiment three times independently.

### 2.3. Colony Formation Assay

The logarithmic growth expectation cells were trypsin digested and suspended in a DMEM medium containing 10% FBS. After cell counting, a six-well plate was inoculated with 1 × 10^3^ cells per well and cultured in a cell incubator for 10–15 days. Before being stained with 0.5% crystal violet (sigma Aldrich, USA), they were fixed with 4% paraformaldehyde once the cells grew into clones visible to the naked eye. Under a microscope (Bethesda, MD, USA), colonies were counted and photographed. Each group is provided with 3 multiple holes.

### 2.4. Transwell Assay

A 24-well insert transwell assay and a Matrigel invasion assay (8.0 *μ*m, Corning, NY, USA) were performed to investigate in vitro cell invasion. Transwell assay was conducted as directed by the manufacturer and as previously described [10]. Briefly stated, Matrigel (50 mg/L, BD, USA) was diluted in the ratio of 1 : 15 before being applied to the upper membrane surface in an amount of 100 L. Subsequently, Matrigel was solidified after 3 h of incubation at 37°C. After being digested and resuspended in a serum-free medium, the cells in the logarithmic phase were adjusted to have a concentration of 5 × 10^5^ cells per milliliter. Then, the upper chamber in a 24-well Transwell plate was supplied with 100 *μ*L suspension and the lower chamber with 600 *μ*L of the 20% serum culture solution. For each well, three replicates were created. Incubation of the transwell inserts took place for 20 hours at a steady 37°C and 5% of CO_2_ in an incubator. After that, the matrix and noninvasive cells were removed from the upper membrane surface using a cotton swab. Subsequently, 4% paraformaldehyde was utilized for fixture of the invasive cells and 0.5% of crystal violet solution (Sigma-Aldrich, USA) for cell staining. The cells were examined under a microscope after washing and drying and the images were collected.

### 2.5. Determination of Reactive Oxygen Species

ROS assay was conducted as instructed by the manufacturer. In brief, the cells were evenly inoculated into a 6-well plate at 1 × 10^5^ cells/well, and different reagents were utilized to treat cells for 24 hours according to the experiment requirements. Then, 0.25% of trypsin without ethylenediaminetetraacetic acid (EDTA) was utilized to digest the treated cells. On completion of digestion, the cells were centrifuged and collected. After washing with PBS three times, 10 *μ*M of dichloro-dihydro-fluorescein diacetate (DCFH-DA) was applied to the cells for incubation at 37°C following three rounds of PBS washing. After 20 min, the cells were resuspended in 500 l of PBS after being washed with serum-free media three times. Cell fluorescence was detected using flow cytometry at wavelengths of 525 nm for excitation and 485 nm for emission. With the results of three replicate wells, the average value was obtained and the specific formula was shown as follows: ROS = fluorescence intensity/(protein concentration × 0.19).

### 2.6. Biochemical Kit-Based Assay

Cells were lysed with RIPA lysis solution (Solarbio, China) on ice after being washed thrice with PBS. Following lysis, the cells were collected into EP tubes. The supernatant was collected for detection after centrifugation at 4°C and 12000 r/min for 30 min. According to the biochemical assay kit (Nanjing Jiancheng Bioengineering Institute, China), Fe^2+^, glutathione (GSH), and malondialdehyde (MDA) levels in the cells were determined. Three independent replications of each experiment were performed.

### 2.7. Western Blot

With the help ofRIPA lysis buffer (Solabio, China), the total protein was extracted from cells and tissues. The concentration of the extracted protein was determined with BCA kit (Beyotime, China), and 20 *μ*g of protein was added to 5× loading buffer to boil for denaturation and denatured using SDS. By using 10% PAGE to separate the proteins, the resulting proteins were transferred to PVDF membranes by membrane transfer. The membranes were prepared by blocking them with 5% nonfat dry milk or 8% BSA (phosphorylated protein) for 2∼3 h, and then mixed with the primary antibody anti-SLC7A11-antibody (1 : 1000, ab175186, Abcam), anti-TRF1-antibody (1 : 1000, ab129177, Abcam), anti-FPN-antibody (1 : 1000, ab235166, Abcam), anti-RAS-antibody (1 : 1000, ab235166, Abcam) 1000, ab52939, Abcam), anti-MEK-antibody (1 : 1000, ab32091, Abcam), anti-p-MEK-antibody (1 : 1000, Abcam-ab96379) anti-ERK-antibody (1 : 10000, M5670, Sigma), anti-pERK-antibody (Thr202/Tyr204) (1 : 1000, 9101S, Cell Signaling), and anti-*β*-actin-antibody (1 : 5000, ab8226, Abcam) were incubated overnight at 4°C. After three TBST washes the next day, the membrane was incubated with secondary antibodies, including goat antimouse IgG (1 : 5000, ab6789, Abcam), goat antirat IgG (1 : 5000, ab97057, Abcam) at ambient temperature, and goat antirabbit IgG (1 : 5000, ab6721, Abcam) for 2 h. ECL chemiluminescence reagent (Solebo, China) was used to display the protein bands, and Image J software to analyze the gray levels of the protein bands. Additionally, the relative protein expression was determined taking *β*-actin as an internal reference.

### 2.8. Statistical Analysis

With the use of SPSS 26.0, statistical analysis was carried out on all data results, which were presented as means with standard deviations (SD). One-way analysis of variance (ANOVA) was employed to determine the significant differences, followed by Dunnett's tests for multiple comparisons or unpaired Student's *t*-tests for two-group comparisons. *P* < 0.05 was deemed significantly different.

## 3. Results

This study sought to dig out the potential use of simvastatin as a chemotherapeutic drug. We hypothesized that simvastatin inhibits Ishikawa cell proliferation, colony formation, and invasion, and promotes cell oxidation and ferroptosis. Therefore, we performed Transwell assays, colony formation, and MTT to detect the effects of different treatments of simvastatin on the invasion, colony formation, and proliferation ability of Ishikawa cells, respectively. Flow cytometry was used to detect intracellular ROS levels; and enzyme linked immunosorbent assay (ELISA) to test intracellular Fe^2+^, MDA, and GSH levels. In addition, the expression level of RAS/mitogen-activated protein kinase (MAPK)-related proteins and ferroptosis-related proteins were detected using Western blot. Our results suggested that simvastatin decreased RAS/MAPK signaling pathway activity and inhibited Ishikawa cell proliferation, colony formation, and invasion, and promoted cellular oxidation and iron ferroptosis. Collectedly, simvastatin has the potential to be a new anticancer drug for EC.

### 3.1. Simvastatin Inhibits the Invasion, Colony Formation, and Proliferation of Ishikawa Cells

To identify the effects of simvastatin on the invasion, proliferation, and other phenotypes of Ishikawa cells, colony formation, MTT, and transwell assays were performed. Relative to the control group, simvastatin treatment could lower the proliferation rate (Figure 1(a)), colony formation (Figures 1(b) and 1(c)), and invasion ability (Figures 1(d) and 1(e)) of Ishikawa cells. The inhibitory effect of simvastatin was dose-dependent; 10 *μ*M and 15 *μ*M groups exhibited more significant inhibitory effect. The above suggested that simvastatin could suppress the invasion, colony formation, and proliferation of Ishikawa cells.

### 3.2. Simvastatin Increases the Oxidation Level of Ishikawa Cells

To observe whether simvastatin affected the oxidation level of Ishikawa cells, flow cytometry and ELISA were utilized to analyze ROS, MDA, and GSH levels in Ishikawa cells receiving different concentrations of simvastatin (5 *μ*M, 10 *μ*M, and 15 *μ*M). The outcome revealed that both 10 *μ*M and 15 *μ*M of simvastatin could increase the ROS level (Figures 2(a) and 2(b)) and MDA level (Figure 2(c)) (*P* < 0.01), but only the latter remarkably decreased the GSH level (Figure 2(d), *P* < 0.01). Additionally, although 5 *μ*M of simvastatin could also increase the level of ROS, MDA, and GSH in cells, no significant differences were observed compared with the control group. The above suggested that simvastatin with high concentration could significantly increase the oxidation level of Ishikawa cells.

### 3.3. Simvastatin Promotes Ferroptosis in Ishikawa Cells

An association between increased ROS levels and cellular ferroptosis has been reported in the literature [21]. Cystine/glutamate antiporter SLC7A11/xCT and ferroportin (FPN) serve as negative regulators of ferroptosis, while TRF1 protein acts as a positive regulator [22]. To clarify whether simvastatin caused ferroptosis in Ishikawa cells, we determined the Fe^2+^ and ferroptosis-related proteins (SLC7A11, TRF 1 and FPN) levels in cells receiving different concentrations of simvastatin. Western blot results displayed that in contrast to the control group, simvastatin could obviously decrease the SLC7A11 and FPN protein expression levels in Ishikawa cells (*P* < 0.01) and increase dose-dependently TRF1 expression (*P* < 0.01) (Figures 3(a)–3(d)). In addition, after treatment with 10 *μ*M and 15 *μ*M of simvastatin, a remarkably dose-dependently increase was observed in the level of Fe^2+^ in cells (Figure 3(e)); while 5 *μ*M of simvastatin had no significant effect on Fe^2+^ level. The above outcomes indicated that simvastatin could promote the ferroptosis in Ishikawa cells.

### 3.4. Simvastatin Inhibits the RAS/MAPK Signaling Pathway in Ishikawa Cells

The RAS/MAPK signaling pathway is responsible for the regulation of cancer initiation and progression, including cell proliferation, differentiation, and survival in a variety of solid and hematological cancers. The overexpression and overactivation of the members of Ras/MAPK cascade have been observed in tumors [23]. For investigating the function of the RAS/MAPK pathway in the Ishikawa cell growth and invasion, related proteins of this pathway (RAS, p-ERK, p-MEK, MEK, and ERK) were detected using Western blot. The results revealed that, simvastatin treatment (10 *μ*M and 15 *μ*M) significantly reduced the RAS, p-MEK, and p-ERK levels, and the ratios of p-MEK/MEK and p-ERK/ERK in a dose-dependent manner (Figures 4(a)–4(d)). Therefore, simvastatin may inhibit the Ishikawa cell proliferation and invasion through the RAS/MAPK signaling pathway.

### 3.5. RAS Agonist Reverses the Inhibitory Effects of Simvastatin on Ishikawa Cell Invasion, Colony Formation, and Proliferation

To further clarify whether simvastatin exerted its inhibitory effect on the Ishikawa cell growth by inhibiting the RAS/MAPK signaling pathway, the invasion, colony formation, and proliferation ability of the cells were detected after treatment with RAS agonist (ML-098) and 15 *μ*M of simvastatin simultaneously. The above malignant behaviors of the cells were significantly promoted in the simvastatin + ML-098 group relative to the simvastatin group (Figures 5(a)–5(e)). Taken together, simvastatin's inhibitory effect on Ishikawa cell invasion, colony formation, and proliferation may be reversed by ML-098 when used in combination.

### 3.6. ML-098 Reverses the Promoting Effects of Simvastatin on Oxidation and Ferroptosis in Ishikawa Cells

Further, we researched the effects of simultaneous ML-098 and simvastatin treatment on oxidative substances (ROS, GSH, and MDA), Fe^2+^ and ferroptosis-related proteins (SLC7A11, TRF 1, and FPN) levels in Ishikawa cells. The investigation results indicated that in contrast to the simvastatin group, the ROS, MDA, and Fe^2+^ levels in cells of simvastatin + ML-098 group were decreased, while GSH level was remarkedly increased (*P* < 0.01, Figures 6(a)–6(e)). In addition, Western blot results suggested that the SLC7A11 and FPN protein levels in the cells of simvastatin + ML-098 group were significantly higher than those in the simvastatin group, while the protein expression level of TRF1 was remarkably lower (Figures (f)6-6(g)). The above suggested that ML-098 could reverse the antitumor effect of simvastatin.

## 4. Discussion

Statins, in addition to lowering cholesterol, can also exert various anticancer effects in liver, colon, and breast cancers, such as antiproliferation, pro-apoptosis, antiangiogenesis, immunoregulation, and anti-invasion [24, 25]. As one of the statins, simvastatin may have potential to treat and prevent cancers. Jin et al. discovered that simvastatin could reduce the viability of EC cells (RL-95-2, Ishikawa and HEC-1B) and induce cell apoptosis [26]. MTOR inhibition may be a mechanism for the antiproliferative actions of simvastatin and metformin, as evidenced by the upregulation of phosphorylated AMPK and the down-regulation of downstream phosphorylated S6 following their treatment [26]. We also found that 10 *μ*M and 15 *μ*M of simvastatin could significantly dose-dependently reduce cell proliferation rate, colony formation, and invasive ability. Long-term exposure to simvastatin can more effectively inhibit the growth of poorly differentiated cells derived from the lung (Calu-3 and Calu6), skin (SCC-M7 and SCC-P9), colon (Caco-2 and HCT-116), prostate (LNCaP and PC-3), breast (MCF7 and SKBr-3) and other tissues [27]. Moreover, simvastatin also has a more significant effect on cells of highly metastatic malignant tumors than it does on cells of benign tumors with the same origin; and this may be related to the need of metastatic tumor cells for more isoprene and mevalonate to improve cell survival [28].

One of the most significant factors contributing to the initiation, metastasis, and progression of cancer is the disruption of redox equilibrium [29]. It is reported that the imbalance of redox homeostasis is caused by increased free radicals (mainly ROS) [21]. Several studies have revealed that a variety of anticancer drugs induce apoptosis and autophagy by generating ROS. For example, resveratrol, a natural polyphenol, regulates antioxidant enzymes to induce mitochondrial H_2_O_2_ accumulation, and then to induce apoptosis of prostate cancer cells PC-3, breast cancer cells MCF-7, and liver cancer cells HepG2 [30]. Existing studies have proved the promotion of simvastatin to ROS production. For instance, Buranrat et al. claimed that simvastatin could significantly promote the accumulation of ROS in MCF-7 cells, so that doxorubicin had a greater effect [31]. Wang et al. pointed out that simvastatin caused an increase of ROS level and then induced apoptosis in OCM-1 cells [32]. In this study, 10 *μ*M and 15 *μ*M of simvastatin could increase the ROS level in Ishikawa cells. Collectively, simvastatin-induced cancer cell death is associated with ROS accumulation.

Ferroptosis is thought to be characterized by lipid peroxidation [33], and ROS-induced lipid peroxidation is a key factor in ferroptosis [21]. At present, cancer treatment regimens based on ferroptosis-induction are effective in reducing the amount of cancer cells. For example, the Food and Drug Administration (FDA) has authorized sorafenib, a medication for the induction of ferroptosis, for the treatment of hepatocellular carcinoma [34]. In this paper, simvastatin could significantly increase the Fe^2+^ level and MDA level, decrease the level of GSH, downregulated the SLC7A11 and FPN levels, and upregulated the TRF1 level. SLC7A11/xCT can promote cystine uptake and glutathione biosynthesis, thereby preventing oxidation and ferroptosis [35, 36]. All in all, simvastatin can exert an anticancer effect by inducing ferroptosis in cells.

Simvastatin suppresses the proliferation of cancer cells by triggering apoptosis and slowing the progression of the cell cycle via a variety of cell signaling pathways, as shown by several in vitro studies. In the measurement of ferroptosis-related proteins, we discovered that simvastatin could greatly promote the TRF1 expression, and some research studies also revealed the correlation of TRF1 expression with the RAS/MAPK pathway activation [37]. Furthermore, the stimulation of the RAS/MAPK pathway can restore the sensitivity of tumor cells to anticancer drugs, which has been presented in many articles [38]. Besides, some other scholars have stated that the sensitivity of ferroptosis in individual cell lines can be determined by the RAS/MAPK pathway [39]. Briefly, one important signaling pathway that controls ferroptosis in cancer cells is the RAS/MAPK pathway. Interestingly, Afrin et al. pointed out that simvastatin could reduce the protein level of RAS and affect the activity of the RAS/MAPK pathway [40]. In this paper, we also discovered that simvastatin inhibited RAS/MAPK pathway activity in Ishikawa cells. For further confirmation, cells were treated with ML-098 (an agonist of the RAS/MAPK pathway) and simvastatin simultaneously, and the outcomes suggest that ML-098 significantly weakened the effects of simvastatin. It could be concluded that simvastatin inhibited the RAS/MAPK signaling pathway to suppress the proliferation, clone formation, invasion of EC cells, and induce ferroptosis.

This study has certain restrictions as well. Firstly, only Ishikawa cells were selected to explore the function and mechanism of simvastatin. However, a study by Kim et al. revealed that simvastatin consistently had an impact on three EC cells (RL-95-2, HEC-1B, and Ishikawa) [26]. So we suspected similar effects of simvastatin in other EC cells as in Ishikawa cells. Besides, Kim et al. also revealed a stronger anticancer effect of the combination of simvastatin and met form than a single drug in their study [26], so further investigation on combined drugs can be performed to obtain better clinical efficacy. Furthermore, only *in vitro* experiments were conducted in our paper, and more comprehensive experimental data are expected to be obtained by further *in vitro* experimental validation.

## 5. Conclusion

To sum up, simvastatin inhibits cell colony formation, invasion, and proliferation in EC Ishikawa cells by suppressing the RAS/MAPK signaling pathway. Besides, the inhibition to the RAS/MAPK signaling pathway allows simvastatin to induce ferroptosis through up-regulating the level of ROS, MDA, Fe^2+^, and TRF1 and reducing the level of GSH, SLC7A11, and FPN in cells. In a word, simvastatin has the potential to be a targeted drug for EC treatment.

## Figures and Tables

**Figure 1:** Simvastatin inhibits the proliferation, colony formation, and invasion of Ishikawa cells. (a): MTT to detect the proliferation of Ishikawa cells treated with simvastatin in different concentrations; (b–c): colony formation assay to measure the clone formation of Ishikawa cells treated with simvastatin in different concentrations; (d–e): transwell to detect the invasion of Ishikawa cells treated with simvastatin in different concentrations, ^*∗*^*P* < 0.01 and ^*∗∗*^*P* < 0.01 vs. control group; ^##^*P* < 0.01 vs. 5 *μ*M group.

**Figure 2:** Simvastatin increases the oxidation level of Ishikawa cells. (a–b): flow cytometry to detect ROS level in Ishikawa cells treated with simvastatin in different concentrations; (c–d): ELISA to detect MDA (c) and GSH (d) levels in Ishikawa cells treated with simvastatin in different concentrations,  ^*∗*^ ^*∗*^*P* < 0.01 vs. control group; ^##^*P* < 0.01 vs. 5 *μ*M group. ROS, reactive oxygen species; MDA, malondialdehyde; GSH, glutathione.

**Figure 3:** Simvastatin promotes ferroptosis in Ishikawa cells. (a–d): Western blot for detection of the effect of simvastatin on the expression of ferroptosis-related proteins (SLC7A11, FPN, and TRF 1) (a) and quantitative analysis based on Image J (b–d); (e): ELISA for detection the effect of simvastatin on Fe^2+^ level in Ishikawa cells, ^*∗∗*^*P* < 0.01 vs. control group; ^##^*P* < 0.01 vs. 5 *μ*M group. SLC7A11, solute carrier family 7 member 11; TRF1, transferrin receptor 1; FPN, ferroportin.

**Figure 4:** Simvastatin inhibits the RAS/MAPK signaling pathway in Ishikawa cells. (a–d): Western blot to detect the effect of simvastatin with different concentrations on the expression of RAS/MAPK pathway-related proteins (RAS, p-MEK, MEK, p-ERK, and ERK) in Ishikawa cells (a), and quantitative analysis based on Image J (b–d), ^*∗*^*P* < 0.05 vs. control group; ^##^*P* < 0.01 vs. 5 *μ*M group.

**Figure 5:** RAS agonist reverses the inhibitory effects of simvastatin on Ishikawa cell proliferation, colony formation, and invasion. (a): MTT assay to detect the effect of simultaneous treatment of ML-098 and simvastatin on the proliferation of Ishikawa cells; (b–c): colony formation assay to explore the effect of simultaneous treatment of ML-098 and simvastatin on the colony formation ability of Ishikawa cells; (d–e): transwell assay to detect the effect of simultaneous treatment of ML-098 and simvastatin on the invasion ability of Ishikawa cells, ^*∗∗*^*P* < 0.01 vs. control group; ^##^*P* < 0.01 vs. simvastatin group.

**Figure 6:** RAS agonist reverses the promoting effects of simvastatin on ROS level and ferroptosis in Ishikawa cells. (a–b): flow cytometry detected the effects of simultaneous treatment of ML-098 and simvastatin on DCFH-DA-labeled ROS level in Ishikawa cells; (c–d): ELISA detected the effects of simultaneous treatment of ML-098 and simvastatin on the level of MDA (c) and GSH (d) in Ishikawa cells; (e): ELISA to detect the effect of simultaneous treatment of ML-098 and simvastatin on the Fe^2+^ level in Ishikawa cells; (f-g): Western blot to determine the effect of simultaneous treatment of ML-098 and simvastatin on the expression of ferroptosis-related proteins (SLC7A11, TRF1, and FPN) in Ishikawa cells, ^*∗∗*^*P* < 0.01 vs. control group; ^##^*P* < 0.01 vs. simvastatin group. ROS, reactive oxygen species; MDA, malondialdehyde; GSH, glutathione; solute carrier family 7 member 11; TRF1, transferrin receptor 1; FPN, ferroportin.

## Data Availability

The data used to support the findings of this study are available from the corresponding author upon request.
